RETRACTED

# Long Non-Coding RNA HOTAIR Regulates the Proliferation, Self-Renewal Capacity, Tumor Formation and Migration of the Cancer Stem-Like Cell (CSC) Subpopulation Enriched from Breast Cancer Cells

**DOI:** 10.1371/journal.pone.0170860

**Published:** 2017-01-25

**Authors:** Jia Deng, Mengchang Yang, Rong Jiang, Ning An, Xiaoshan Wang, Bin Liu

**Affiliations:** 1 Department of Anesthesiology, West China Hospital, Sichuan University, Chengdu, Sichuan, P.R. China; 2 Department of Anesthesiology, Sichuan Academy of Medical Sciences and Sichuan Provincial People’s Hospital, Chengdu, Sichuan, P.R. China; 3 Department of oncology, Sichuan Academy of Medical Sciences and Sichuan Provincial People’s Hospital, Chengdu, Sichuan, P.R. China; University of South Alabama Mitchell Cancer Institute, UNITED STATES

## Abstract

**Purpose:**

Long non-coding RNAs (lncRNAs) play important roles in the malignant behavior of cancer. HOTAIR, a well-studied lncRNA, contributes to breast cancer development, and overexpression of HOTAIR predicts a poor prognosis. However, the regulatory role of HOTAIR in the cancer stem-like cell (CSC) subpopulation remains largely unknown. Our goal was to determine the regulatory functions of HOTAIR in the processes of self-renewal capacity, tumor formation and proliferation of CSCs derived from breast cancer.

**Methods:**

We first enriched and incubated the CSC population derived from breast cancer cell line MCF7 (CSC-MCF7) or MDA-MB-231 (MB231, CSC-MB231). Self-renewal capacity and tumor formation were assessed in vitro and in vivo to determine the stemness of CSCs. We assessed the impact on ectopically upregulated or downregulated expression of HOTAIR in CSCs by soft agar, self-renewal capacity and CCK-8 assays. The functional domain of HOTAIR was determined by truncation. RT-qPCR and semiquantitative Western blotting were performed to detect the expression levels of genes of interest. Chromatin IP (ChIP) was employed to detect the transcriptional regulatory activity of p53 on its target gene.

**Results:**

After the identification of CSC properties, RT-qPCR analysis revealed that HOTAIR, but not other cancer-associated lncRNAs, is highly upregulated in both CSC-MCF7 and CSC-MB231 populations compared with MCF7 and MB231 populations. By modulating the level of HOTAIR expression, we showed that HOTAIR tightly regulates the proliferation, colony formation, migration and self-renewal capacity of CSCs. Moreover, full-length HOTAIR transcriptionally inhibits miR-34a specifically, leading to upregulation of Sox2, which is targeted by miR-34a. Ectopic introduction of miR-34a mimics reverses the effects of HOTAIR on the physiological processes of CSCs, indicating that HOTAIR affects these processes, including self-renewal capacity; these effects are dependent on the regulation of Sox2 via miR-34a. Interestingly, tight transcriptional regulation of p53 by HOTAIR was found; accordingly, p21 is indirectly regulated by HOTAIR, resulting in cell cycle entry.

RETRACTED

**Conclusion:**

These results suggest that HOTAIR is a key regulator of proliferation, colony formation, invasion and self-renewal capacity in breast CSCs, which occurs in part through regulation of Sox2 and p53.

## Introduction

lncRNAs, which are typically non-protein coding transcripts longer than 200 nucleotides, can epigenetically interact with transcription factors, transcriptional activators or repressors, and different subunits of complexes, including RNA polymerase (RNAP) II and even duplex DNA, to function as transcriptional or post-transcriptional regulators [1]. As a result of their regulatory roles, lncRNAs strongly influence the malignant behavior of cancer, such as tumorigenesis, proliferation, apoptosis, chemoresistance and invasiveness [1]. For example, metastasis-associated lung adenocarcinoma transcript 1 (MALAT-1), an evolutionarily highly conserved and ubiquitously expressed lncRNA, is reportedly highly upregulated in several human malignancies in addition to lung cancer, and it was found to be tightly associated with clinical parameters and promoted invasion and metastasis [2]. However, the functions of thousands of lncRNAs are still unknown, and the extent of their involvement in tumorigenesis is only beginning to be understood.

HOTAIR (Hox transcript antisense intergenic RNA), an approximately 2.2 kb-long non-coding RNA transcribed from the HOXC locus, epigenetically functions as a repressor of HOXD [3]. A novel molecule in the field of tumor biology, HOTAIR has been correlated with metastasis in a variety of cancer types, including colorectal [4], pancreatic [5], lung [6] and breast [7] cancers. Notably, a study of its regulatory mechanism in breast cancer revealed that HOTAIR promotes breast cancer metastasis, partly by interacting directly with polycomb repressive complex-2 (PRC2) through its 5’ domain to induce genome-wide retargeting of PRC2 to hundreds of genes involved in metastasis. The result is H3K27 methylation, which epigenetically silences these genes [7]. Moreover, HOTAIR directly inhibits WIF-1 expression by promoting H3K27 methylation in the responding promoter region, thereby activating Wnt/β-catenin signaling [8]. Accordingly, HOTAIR plays key roles in the epigenetic regulation of breast cancer malignancy.

Breast cancer is one of the most common diseases in females, and several novel therapeutics have been developed thus far. Nonetheless, metastasis remains poorly understood, is largely incurable, and is the main cause of cancer-related death [9]. Recently, the cancer stem-like cell (CSC) hypothesis has provided new insight into tumorigenesis and metastatic progression, potentially explaining the metastatic mechanisms of breast cancer. This hypothesis suggests that breast CSCs, a subpopulation of breast cancer cells, but not the original tumor cells are responsible for tumor development, metastasis, and transplantation processes [10]. In original breast cancer cells, metastasis appears to be tightly controlled by MALAT-1 expression, which is upregulated by 17β-estradiol treatment [11]. Nonetheless, the functions of lncRNA in breast CSCs are unknown.

RETRACTED

Accumulated evidence has revealed that interaction of lncRNA with DNA, RNA, and proteins affects all levels of gene regulation, including chromatin remodeling, transcription, pre-mRNA splicing, mRNA turnover, mRNA translation, and protein stability [12–15]. HOTAIR is reported to directly interact with microRNA-34a (miR-34a) [16], which in turn downregulates expression of HOTAIR in prostate cancer (PCa) cell lines by binding to the mRNA. Interestingly, Liu et al. found that HOTAIR epigenetically represses miR-34a by enhancing DNA methylation of the promoter region [17]. Taken together, HOTAIR and miR-34a form a feedback-loop that achieves a dynamic balance of their regulatory effects on physiological processes.

p53 functions in response to a variety of cellular stress signals to induce cell cycle arrest and thus decrease cell proliferation and promotes cell death [18]. p21, a potent cyclin-dependent kinase inhibitor, is one of its most well-studied downstream target genes. Activated p21 arrests the cell cycle at G1 phase by inhibiting CDK1, CKD2 and CDK4/6 [19]. New clinical research indicates that activation of p53/p21 is strongly associated with poor prognosis in breast cancer patients, and the potential mechanism was further verified in the breast cancer cell line MCF7 [20]. However, the regulatory role of p53/p21 in the proliferation of CSCs remains unclear.

Therefore, in this study, we focused on the expression pattern of HOTAIR in CSCs derived from breast cell lines and examined how interaction between HOTAIR and miR-34a affects the malignant behavior of these CSCs.

## Material and Methods

### Cell cultures

Human breast cancer cell lines MCF7 and MB231 were frozen in our laboratory in liquid nitrogen and cultured in minimal essential medium (MEM) supplemented with 10% fetal bovine serum (FBS), 100 μg/ml penicillin, and 100 μg/ml streptomycin in a 5% CO_2_ incubator at 37°C. To enrich the CSC subpopulation from MCF7 (CSC-MCF7) or MB231 (CSC-MB231) lines, cells were maintained in serum-free medium (SFM) containing DMEM/Ham Nutrient Mixture F-12 (1:1) with the addition of epidermal growth factor (EGF, 20 ng/ml), human fibroblast growth factor basic (hFGFb, 10ng/ml), and 2% B-27 for 14–21 days. The SFM was replaced every 3 days after mild centrifugation of the spheres.

RETRACTED

### Reverse-transcriptional quantitative PCR (RT-qPCR)

Total RNA was extracted using Trizol (Life Technologies, Grand Island, NY, USA) according to the manufacturer’s instructions. For RT-qPCR analysis, 1 μg of total RNA was reverse-transcribed using an RT kit (Life Technologies, Grand Island, NY, USA), and the cDNA was used as the template under the following conditions: 40 cycles of 95°C for 30 s; 55°C for 30 s; and 72°C for 1 min. An ABI7500 (Applied Biosystems, Foster City, CA, USA) was used for qPCR. The primers used for qPCR were as follows: MALAT-1 forward, 5’-GACTTCAGGTCTGTCTGTTCT-3’, and reverse, 5’-CAACAATCACTACTCCAAGC-3’; HOTAIR forward, 5’-GCTTCTAAATCCGTT-3’, and reverse, 5’-CTCCACGGTAAATCCGGCAG-3’; HN forward, 5’-CAGCAAGACGAGAAGACCCT-3’, and reverse, 5’- CCCTAGGGTAACTTGTTCCGT-3’; HIF1A-AS1 forward, 5’-GTCACGATTCGGTACAC-3’, and reverse, 5’-CGCGCAGGTCATAAGAGTTGTG-3’; Bmi1 forward, 5’- CCACCTGATGTGTGTGCTTTG-3’, and reverse, 5’-TTCAGTAGTGGTCTGGTCTTGT-3’; β-catenin forward, 5’- AAAGCGGCTGTTAGTCACTGG-3’, and reverse, 5’-CGAGTCATTGCATACTGTCCAT-3’; c-Myc forward, 5’-GGCTCCTGGCAAAAGGTCA-3’ and 5’- CTGCGTAGTTGTGCTGATGT-3’; Nanog forward, 5’-TTTGTGGGCCTGAAGAAAACT-3’, and reverse, 5’-AGGGCTGTCCTGAATAAGCAG-3’; Sox2 forward, 5’- GCCGAGTGGAAACTTTTGTCG-3’, and reverse, 5’-GGCAGCGTGTACTTATCCTTCT-3’; Oct4 forward, 5’-CTGGGTTGATCCTCGGACCT-3’, and reverse, 5’-CCATCGGAGTTGCTCTCCA-3’. For miRNA qPCR, the results were normalized to U6 expression using U6 forward, 5’-CTCGCTTCGGCAGCACA-3’, and reverse, 5’-AACGCTTCACGAATTTGCGT-3’. The qPCR results were analyzed, and the results are expressed relative to CT (threshold cycle) values. The values were then converted to fold changes, with a fold change of 2.0 considered significant.

### qPCR for miRNA

Levels of miRNA expression were detected by RT-qPCR using a Taqman^®^ MicroRNA assay with the following sequences: miR-16 (Assay ID: 000391, target sequence: 5’ UAGCAGCACGUAAAUAUUGGCG-3’); miR-29b (Assay ID: 000413, target sequence: 5’-UAGCACCAUUUGAAAUCAGUGUU-3’); miR-34a (Assay ID: 002316, target sequence: 5’-CAAUCAGCAAGUAUACUGCCCU-3’); miR-34c (Assay ID: 000428, target sequence: 5’-AGGCAGUGUAGUUAGCUGAUUGC-3’); miR-375 (Assay ID: MC10327, target sequence: 5’-UUUGUUCGUUCGGCUCGCGUGA-3’); miR-101 (Assay ID: 003353, target sequence: 5’-UACAGUACUGUGAUAACUGAA-3’). The qPCR results were analyzed, and the results are expressed relative to CT (threshold cycle) values. The values were then converted to fold changes, with a fold change of 2.0 considered significant.

RETRACTED

### HOTAIR expression and shRNA constructs

The coding sequence of HOTAIR was cloned using the primers HOTAIR-F: 5’-CATGGATCCACATTCTGCCCTGATTTCCGGAACC-3’ and 5’-ACTCTCGAGCCACCACACACACACAACCTACAC-3’ and inserted into the retroviral vector Plvx-EF1α-IRES-Puro (Life Technologies, Grand Island, NY, USA). HOTAIR shRNA vectors (GV248, HOTAIR-shRNA and control shRNA) were purchased from RIBOBIO (Guangzhou, China). 293T cells were transfected with lentivirus expressing shControl, shHOTAIR, or HOTAIR for lentiviral packaging.

### miR-34a mimics and transfection

Two synthetic, chemically modified short single-stranded RNA oligonucleotides (miR-34a mimics and scrambled mimics) were purchased from Life Technologies (Grand Island, NY, USA). Oligonucleotide transfection was performed using X-tremeGENE siRNA Transfection Reagent (Roche) following the manufacturer’s protocol.

### Serial replating assay

Target cells were counted and suspended in SFM supplemented with human growth factors and B-27, as described above. In total, 1,000 cells were plated in SFM supplemented with EGF, bFGF and B27. Colonies were counted on day 7. Cells were harvested and counted, and 1,000 cells were replated for secondary and tertiary rounds. For each round, colonies were counted on day 7.

### Cell migration assay

Cells (5×10^4^) were suspended in 500 μl DMEM medium without FBS and seeded in upper chambers, and 500 μl DMEM containing 10% FBS was added to the lower chamber. After 24 h, the cells were fixed and stained for imaging.

### Cell proliferation assay

Cells were cultured at a density of 5×10^3^ cells per well in a 24-well plate. Cholecystokinin octapeptide (CCK-8) was applied, and cell viability was assessed by measuring the absorbance at 450–620 nm. All assays were performed in triplicate and independently repeated three times.

### Soft agar colony formation assay

To analyze colony formation ability, a total of 1×10^3^ or 1×10^4^ cells was added to 3 ml DMEM supplemented with 10% FBS and mixed with 0.3% agarose (low melt, Bio-Rad, Hercules, CA, USA). The plates were placed at 37°C with high humidity and 5% CO_2_. Colonies were stained and counted after 21 days of growth.

### Tumor growth in NOD-SCID mice

Four to six-week-old male NOD-SCID mice were purchased from Sichuan Dashuo Laboratory (Chengdu, Sichuan, China). All experiments involving live animals were strictly carried out according to the relevant national and international guidelines, as approved by the Medical ethics committee of Sichuan University, West China Hospital. The mice were anesthetized using an intraperitoneal (i.p.) injection of 100 mg/kg ketamine and 5 mg/kg xylazine. In total, 1000 and 10,000 single MCF7 or MB231 cells were suspended in chilled phosphate-buffered saline (PBS) and injected subcutaneously into the right midabdominal area. The tumor sizes were recorded on days 17, 27, 28, and 32 using Vernier calipers. Mice were sacrificed after 32 days.

RETRACTED

### Statistical analysis

All data are presented as the mean with the standard deviation (SD) or median with the 95% confidence interval (95% CI). Statistic comparison was performed using Student’s t-test and one-way ANOVA analysis using SPSS (version 16) software (IBM, Armonk, NY, USA).

## Results

### HOTAIR is overexpressed in CSC-MCF7 or CSC-MB231 populations

As a subpopulation of breast cancer cells, CSCs exhibit significant differences in comparison with the breast cancer cells from which they are derived. One difference involves lncRNA expression, which is reported to be tightly associated with the malignant behavior of breast cancer [14]. To determine differences in the expression of lncRNAs between CSCs and breast cancer cells, CSCs were first enriched from MCF7 or MB231 cells. As is characteristic of CSCs, the formation of spheres was observed after 5 days of culturing in SFM (Fig 1A). On day 17, the sphere diameter reached approximately 100 μM, representing a stage of vigorous growth. As CSCs enriched from cancer cells are presumed to possess high tumor formation capacity, we then separately confirmed the colony formation and tumor formation of the enriched CSC-MCF7 or CSC-MB231 populations. In an in vitro colony formation assay, a small number of CSC-MCF7 or CSC-MB231 (10^3^ cells per well) formed colonies on soft agar, whereas no observable colony was found in the wells in which MCF7 or MB231 cells were seeded (Fig 1B & 1C). In a tumor formation assay, as expected, 1000 and 10000 single CSC-MCF7 or CSC-MB231 cells formed tumors, though the original cells failed to form a visible tumor (Fig 1D). We then performed RT-qPCR to detect the relative levels of MALAT-1, HOTAIR, HN1 and HIF1A-AS expression in CSC-MCF7 or CSC-MB231 compared to MCF7 or MB231. Remarkable upregulation of both MALAT-1 and HOTAIR was found in the CSC-MCF7 and CSC-MB231 populations, especially HOTAIR (Fig 1E).

**Fig 1:** The level of HOTAIR expression in CSC-MCF7 and CSC-MB231 populations. (A) Enrichment of CSC subpopulations from MCF7 and MB231 cells were incubated and photographed on day 5 and day 17. (B) Colony formation by CSCs and their original cells on soft agar when seeded at 10^3^ cells per well or 10^4^ cells per well. (C) Colonies in each well were counted after staining with 0.05% crystal violet. (D) Tumor formation ability of CSCs or their original cells at different amounts was measured in mice, and the tumor volumes were measured from day 10 to day 32. (E) RT-qPCR measurement of the expression levels of MALAT-1, HOTAIR, HN-1 and HIF1A-AS in CSC-MCF-7 or CSC-MB231. *P<0.05.

RETRACTED

### HOTAIR expression regulates proliferation, colony formation, migration and self-renewal capacity in CSC- MCF7

HOTAIR is reportedly upregulated in several types of cancers, including breast cancer, and this promotes migration and invasion via induction of the epithelial-mesenchymal transition (EMT). This led us to focus on the effects of upregulated HOTAIR in breast CSCs. CSC-MCF7 and CSC-MB231 presented a similar cellular phenotype; thus, CSC-MCF7 was employed for the ensuing analysis. First, a lentivirus vector expressing HOTAIR (LV-HOTAIR) or shRNA targeting HOTAIR (LV-HOTAIR^KD^) was constructed; a lentivirus vector expressing scrambled shRNA (LV-scrambled) was used as the negative control. To confirm the infection efficiency, the lentiviruses were incubated with unattached CSC-MCF7 spheres in a 24-well plate. After 72 h, the enhanced green fluorescent protein (eGFP) signal was detected after 4',6-diamidino-2-phenylindole (DAPI) staining of nuclei (Fig 2A). The results indicated successful infection. We then tested the effects of HOTAIR on proliferation, colony formation, migration and self-renewal capacity in CSC-MCF7. Overexpression of HOTAIR significantly promoted CSC-MCF7 proliferation (Fig 2B), colony formation (Fig 2C) and migration (Fig 2D)compared with the negative control (LV-vector). As expected, when HOTAIR was knocked down LV-HOTAIR^KD^, inhibition of proliferation (Fig 2B), colony formation (Fig 2C), migration (Fig 2D) and self-renewal capacity (Fig 2E) of CSC-MCF7 was observed, indicating a direct association between HOTAIR and these cellular physiological processes. Furthermore, examination of the percentages of cell cycle distribution by propidium iodide (PI) staining-based fluorescence-activated cell sorting (FACS) analysis confirmed that the cell proliferation due to HOTAIR is caused by promotion of cell cycle transition from G0-G1 to S phase (Fig 2F).

**Fig 2:** Expression of HOTAIR in CSC-MCF7 regulates proliferation, colony formation, migration and self-renewal capacity. (A) Detection of eGFP confirmed the successful infection of LV-HOTAIR or LV-HOTAIR^KD^. (B) A CCK-8 assay was performed to detect proliferation in MCF7 cells transfected with LV-HOTAIR, LV-scrambled or LV-HOTAIR^KD^. (C) A colony formation assay was performed in MCF7 cells transfected with LV-HOTAIR, LV-scrambled or LV-HOTAIR^KD^ (Left panel); the colonies in each well were counted after nitro blue tetrazolium (NBT) staining (Right panel). (D) A migration assay was performed in uncoated transwell chambers (Left panel); the cells that migrated through the membrane were stained with 0.05% crystal violet and counted (Right panel). (E) Self-renewal capacity was detected in serum-free medium; spheres (>40 μm in diameter) were counted per well at different passages. *P<0.05.

RETRACTED

### Overexpression of HOTAIR attenuates miR-34a to achieve effects on cellular physiological processes

Accumulated evidence shows that lncRNAs potentially regulate other classes of non-coding RNAs, especially miRNAs. To investigate the effect of HOTAIR on potential downstream miRNAs, six miRNAs highly enriched downstream of HOTAIR were chosen and detected in CSC-MCF7 and MCF7 cells. By performing RT-qPCR, we found that miR34a expression was upregulated in CSC-MCF7 or CSC-MB231 cells (Fig 3A). We then ectopic expressed or knocked down HOTAIR in CSC-MCF7 cells and assessed the effect of changes in HOTAIR expression on miR-34a. According to the results, miR-34a was significantly affected, without changes in other miRNAs (Fig 3B). To determine the site responsible for HOTAIR’s impact on miR-34a expression, full-length HOTAIR was truncated as described in Fig 3C. The effect of full-length HOTAIR and the five truncations on miR-34a and miR-34c were examined after transfection for 48 h. Interestingly, only transfection with full-length HOTAIR, and not any of the five truncations, notably affected miR-34a expression, suggesting that full-length HOTAIR is required for miR-34a regulation (Fig 3D). We then introduced antago-miR-34a into CSC-MCF7 cells to compare the effects of HOTAIR overexpression with the direct inhibition of miR-34a. As expected, similar effects on proliferation were observed (Fig 3E). To further confirm the association of HOTAIR with miR-34a, we co-transfected LV-HOTAIR and miR-34a mimics into CSC-MCF7 and found that overexpression of HOTAIR was attenuated by miR-34a mimics (Fig 3F).

**Fig 3:** Expression of HOTAIR transcriptionally inhibits expression of miR-34a. (A) The levels of miR-16, miR-29b, miR-34a, miR-34c, miR-375 and miR-101 expression were detected in CSC-MCF7 or CSC-MB231 by RT-qPCR. (B) After transfection of LV-scrambled, LV-HOTAIR^KD^, or LV-HOTAIR into CSC-MCF7 cells, the miRNAs mentioned above were detected by RT-qPCR. (C) HOTAIR truncations were cloned. (D) After the transfection of the truncations, the levels of miR-34a and miR-34c in transfected CSC-MCF7 cells were detected by RT-qPCR. (E) For comparison of the effect of HOTAIR and miR-34a on proliferation, CCK-8 assays were performed in these transfected cells. (F) After co-transfection of LV-HOTAIR with miR-34a mimics or scrambled mimics, CCK-8 assays were performed. *P<0.05, **P<0.01.

RETRACTED

### HOTAIR regulates the self-renewal capacity of CSC-MCF7 by affecting Sox2 via transcriptional regulation of miR-34a

Considering the above results showing the primary effects of HOTAIR on invasion, self-renewal capacity and tumor formation, we tested expression of specific genes strongly associated with these processes. The RT-qPCR results showed that β-catenin, which is associated with EMT promotion, is tightly regulated by HOTAIR expression (Fig 4A). In addition, Sox2, a key transcriptional factor that regulates self-renewal maintenance, was positively regulated by HOTAIR overexpression (Fig 4A). Therefore, we focused on whether the effect of HOTAIR overexpression on Sox2 occurs through direct regulation of miR-34a by transfecting LV-HOTAIR/miR-34a mimics into CSC-MCF7 cells. As expected, transfection of LV-HOTAIR or LV-HOTAIR/scrambled mimics significantly upregulated Sox2 mRNA and protein levels (Fig 4B left and right panels), whereas co-transfection of LV-HOTAIR and miR-34a mimics caused no detectable change in Sox2 mRNA and protein levels. These findings indicate that HOTAIR tightly regulates Sox2expression and that this regulation can be disturbed by epigenetic expression of miR-34a. To further confirm the effect of HOTAIR on self-renewal capacity and tumor formation via regulation of Sox2 expression through miR-34a, self-renewal capacity and colony formation assays were performed after the above-mentioned co-transfection (Fig 4B). Consistent with previous observations, epigenetic expression of HOTAIR by LV-HOTAIR transfection promoted self-renewal capacity and colony formation compared with the negative control (CSC-MCF7 transfected with the LV vector) (Fig 4C and 4D). Co-transfection of LV-HOTAIR and miR-34a mimics resulted in no remarkable change in self-renewal capacity or colony formation (Fig 4C and 4D).

**Fig 4:** HOTAIR regulates the Sox2 expression via miR-34a and affects CSC self-renewal capacity. (A) The levels of Bmi1, β-catenin, c-Myc, Nanog, Sox2 and Oct4 expression in CSC-MCF7 cells transfected with LV-HOTAIR^KD^, LV-scrambled or LV-HOTAIR were detected by RT-qPCR. (B) The mRNA levels (Left panel) and protein levels (right panel) of Sox2 in CSCs were analyzed by RT-qPCR and semi-quantitative Western blotting. (C) To detect the effects of HOTAIR or miR-34a on CSC self-renewal capacity, a sphere formation assay was performed. (D) To detect the effects of HOTAIR or miR-34a on colony formation, a soft agar assay was performed in which the colonies per well were counted. *P<0.05.

RETRACTED

### Upregulated HOTAIR regulates proliferation and colony formation through the p53/p21 pathway by inducing expression of p53 in CSC-MCF7 cells

Considering the observed induction of cell cycle entry and proliferation promotion via overexpression of HOTAIR (Fig 2B and 2C), we examined the effects of HOTAIR on the p53/p21 pathway. We compared the mRNA and protein levels of p53 and p21 in the original cancer cells and in the CSC-MCF7 or CSC-MB231 population. We found that both p53 and p21 were dramatically downregulated in the CSC subpopulations, which may be the reason for the promotion of proliferation and cell cycle entry (Fig 5A). To further identify the regulatory role of HOTAIR with regard to the p53/p21 pathway, the expression level of HOTAIR was modified in CSC-MCF7 cells by inducing ectopic expression or shRNA-mediated knockdown using a lentiviral vector (Fig 5B). Knockdown of HOTAIR significantly increased the mRNA and protein expression levels of p53/p21, though upregulation of HOTAIR had no detectable effects on p53/p21, indicating partial regulation of HOTAIR on p53/p21. Because of the weak effect observed in the CSC-MCF7 population, MCF7 cells were used to determine the effects of HOTAIR upregulation on p53/p21. The results showed that introduction of HOTAIR dramatically reduced the binding of p53 to the p21 promoter region (Fig 5C). Furthermore, the effect of p53 was achieved through DNA binding activity, acting as a transcriptional regulator of its target downstream genes, including p21 (Fig 5D), which resulted in suppression of proliferation (Fig 5E). To further evaluate the effects of the DNA binding activity of p53 on proliferation and colony formation, PFTα, a specific DNA-binding inhibitor of p53, was added to the cells. As expected, abolishing the DNA binding activity of p53 attenuated the suppression of proliferation and colony formation (Fig 5F and 5G).

**Fig 5:** HOTAIR modifies the p53/p21 pathway and thus regulates CSC proliferation and colony formation. (A) RT-qPCR and semi-quantitative western blotting were applied to detect the mRNA and protein levels of p53 and p21 in original or CSC-MCF7 and CSC-MB231 cells. (B) After introduction of HOTAIR or shRNA targeting HOTAIR into CSCs, expression of p53 and p21 was detected. (C and D) A ChIP assay was performed to detect the binding of native p53 in MCF7 cells (C) or ectopic expressed Flag-P53 in CSCs (D) to the p21 promoter region. (E) A CCK-8 assay to detect CSC-MCF7 cells transfected with Flag-p53^R248Q^ or Flag-p53. (F and G) CCK-8 (F) and colony formation (G) assays to detect the proliferation rate of CSC-MCF7-LV-HOTAIR with p53 reintroduction and co-culture with 30 μM PFTα. *P<0.05.

RETRACTED

## Discussion

CSCs are defined as a small fraction of multipotent cells within a tumor that exhibit self-renewal capability and asymmetric cell division [11, 21]. Accumulated evidence has revealed the critical role of CSCs in cancer aggressiveness, metastasis, recurrence and resistance to chemotherapy in several types of cancers. lncRNAs are also reported to play a critical role in cancer progression and metastasis, and one such lncRNAs, HOTAIR, has attracted much attention due to its heightened expression in cancer tissues. For example, in lung cancer and renal cell carcinoma, upregulation of HOTAIR was clearly associated with larger tumor size, advanced pathological stage and extensive metastasis [4, 22, 23, 24]. Overexpression of HOTAIR not only affects tumor formation but also promotes proliferation, migration and invasion in several types of cancers, including gastric, endometrial and lung cancers [9, 25, 26, 27]. The strong association between HOTAIR expression and cancer led us to address whether upregulation of HOTAIR controls cancer by regulating CSCs.

The data from our study suggest that HOTAIR is significantly upregulated in CSC-MCF7 and CSC-MB231 populations. Indeed, expression of HOTAIR is critical for migration, invasion and self-renewal capacity in CSCs enriched from breast cancer cells. Using loss- and gain-of-function experiments, CSC proliferation, self-renewal and migration were found to be regulated by lncRNA [28]. For instance, in CD133-positive CSCs derived from osteosarcoma cells, overexpression of HIF2PUT significantly decreased the CSC population of MG63 cells [11]. Our study found that HOTAIR has a similar role in CSCs derived from breast cancer cells.

Overexpression of HOTAIR in epithelial cancer cells activates the retargeting processes of polycomb repressive complex 2 (PRC2), leading to altered histone H3 lysine 27 methylation and consequent gene expression [7]. Interestingly, genome-wide retargeting of PCR2 has different effects depending on the gene involved. In hepatocellular carcinoma cells, upregulation of HOTAIR promotes migration and invasion by inhibiting RBM38 while activating the Wnt/β-catenin pathway [29, 30]. However, in our study, we did not detect inhibition of RBM38 or activation of Wnt/β-catenin signaling in CSCs when overexpressing HOTAIR (data not shown). This suggests that other regulatory mechanisms of migration and invasion are affected by HOTAIR in unknown ways.

To understand this, we examined interaction between HOTAIR with DNA, RNA and proteins and finally focused on its interaction with miRNA. Chiyomaru et al. showed that upregulated miR-34a binds directly to HOTAIR mRNA and impacts its expression [16]. Interestingly, Liu et al. revealed the indirect regulatory function of HOTAIR on miR-34a expression by activating the retargeting processes of PRC2 [17]. To test the dynamic balance between HOTAIR and miR-34a, we detected miR-34a expression in CSCs enriched from breast cancer cells and CSCs infected with LV-HOTAIR (Fig 3A and Fig 4A). As expected, the change in HOTAIR expression negatively regulated miR-34a. However, we failed to observe HOTAIR downregulation after introducing miR-34a mimics (data not shown). To search for the functional region of HOTAIR responsible for regulating miR-34a expression, we truncated HOTAIR (Fig 3C) and separately delivered these truncations into CSCs. Except for full-length HOTAIR, all of the truncations failed to affect miR-34a expression, suggesting that the complete HOTAIR sequence is required for it to perform its regulatory role.

RETRACTED

It is generally thought that SOX2, OCT4 and Nanog are key transcriptional regulators that maintain the self-renewal capacity of CSCs [31]. Accumulated data indicate that stable changes in expression of SOX2, OCT4 and Nanog affect self-renewal capacity and, consequently, lead to changes in proliferation, migration and invasion. This prompted us to explore the regulatory role of upregulated HOTAIR on the expression levels of SOX2, OCT4 and Nanog. It has been reported that miR-34a directly targets Sox2 mRNA and reduces its protein level [32]; therefore, we evaluated the level of Sox2 mRNA. As expected, we found that upregulated HOTAIR had a significant effect on SOX2 mRNA. However, no detectable effect on OCT4 or Nanog was observed. The results show that introduction of antago-miR-34a into CSCs had effects on proliferation that were similar to those observed after introduction of HOTAIR. In addition, introduction of miR-34a mimics together with HOTAIR diminished HOTAIR’s effect on proliferation, which further confirmed that the functional role of HOTAIR depends on regulation of miR-34a (Fig 3E).

In summary, our findings first show that upregulation of HOTAIR in CSCs enriched from breast cancer cells might play a critical role in maintaining self-renewal capacity by regulating miR-34a and, consequently, Sox2. We also postulate that CSCs expressing higher levels of HOTAIR could represent more malignant cells. These findings may explain the clinical behavior of CSCs in breast cancer and could provide valuable therapeutic targets.
